The article "Protective Effect of Nicorandil on Cardiac Microvascular Injury: Role of Mitochondrial Integrity" was retracted in 2023. Reasons: signs of a paper mill; suspected computer-generated content; unreliable results or conclusions; concerns about the data.

# Protective Effect of Nicorandil on Cardiac Microvascular Injury: Role of Mitochondrial Integrity

**DOI:** 10.1155/2021/4665632

**Published:** 2021-07-03

**Authors:** Xiaosi Jiang, Dan Wu, Zichao Jiang, Weiwei Ling, Geng Qian

**Affiliations:** ^1^Department of Cardiology, The First Medical Center, Chinese PLA General Hospital, Beijing, China; ^2^School of Medicine, Nankai University, Tianjin, China

## Abstract

A major shortcoming of postischemic therapy for myocardial infarction is the no-reflow phenomenon due to impaired cardiac microvascular function including microcirculatory barrier function, loss of endothelial activity, local inflammatory cell accumulation, and increased oxidative stress. Consequently, inadequate reperfusion of the microcirculation causes secondary ischemia, aggravating the myocardial reperfusion injury. ATP-sensitive potassium ion (K_ATP_) channels regulate the coronary blood flow and protect cardiomyocytes from ischemia-reperfusion injury. Studies in animal models of myocardial ischemia-reperfusion have illustrated that the opening of mitochondrial KATP (mito-K_ATP_) channels alleviates endothelial dysfunction and reduces myocardial necrosis. By contrast, blocking mito-K_ATP_ channels aggravates microvascular necrosis and no-reflow phenomenon following ischemia-reperfusion injury. Nicorandil, as an antianginal drug, has been used for ischemic preconditioning (IPC) due to its mito-K_ATP_ channel-opening effect, thereby limiting infarct size and subsequent severe ischemic insult. In this review, we analyze the protective actions of nicorandil against microcirculation reperfusion injury with a focus on improving mitochondrial integrity. In addition, we discuss the function of mitochondria in the pathogenesis of myocardial ischemia.

## 1. Introduction

Acute myocardial infarction (AMI), as a coronary artery disease, is increasingly becoming a leading cause of death worldwide. In clinical practice, primary percutaneous coronary intervention (PCI) is a standard therapeutic strategy to open blocked vessels in patients with ST-segment elevation myocardial infarction (STEMI), since it shortens the total ischemic time and reduces the mortality rate. However, a few patients still suffer from myocardial postischemic injury, which is termed as the no-reflow phenomenon during or after PCI [1–4]. The potential mechanism of no-reflow phenomenon involves coronary microvascular dysfunction (CMD) which has been considered as an independent risk factor for rehospitalization and 30-day mortality in AMI patients during or after PCI therapy [5]. CMD is often responsible for angina and poor prognosis after PCI in AMI patients [6].

Recently, several researches have confirmed that mitochondrial dysfunction is a key factor in the pathogenesis of AMI and no-reflow phenomenon [7, 8]. Mitochondria maintain microcirculation function by modifying the postischemic injury signals—clearing the damaged mitochondria via mitochondrial autophagy (mitophagy), transmitting the extracellular signals to endothelial cells, and controlling endothelial apoptosis or survival [9–11]. Thus, mitochondrial dysfunction is a characteristic feature of myocardial ischemia-reperfusion injury (IRI) [12–15].

The article "Protective Effect of Nicorandil on Cardiac Microvascular Injury: Role of Mitochondrial Integrity" was retracted in 2023. Reasons: signs of a paper mill; suspected computer-generated content; unreliable results or conclusions; concerns about the data.

Nicorandil is an antianginal drug with nitrate-like effects. It exerts its cardiomyocyte protection effects by directly opening the mitochondrial ATP-sensitive potassium ion (KATP) channels, increasing the K^+^ influx, depolarizing the mitochondrial membrane, blocking mitochondrial Ca^2+^ uptake, restoring mitochondrial function, promoting ATP generation, alleviating ischemic damage, and preventing cardiomyocyte apoptosis [16, 17] (Table 1). Nicorandil's core property of maintaining mitochondrial integrity makes it a suitable candidate for inhibiting microcirculatory reperfusion injury.

## 2. Pathophysiological Mechanisms of Microcirculatory Reperfusion Injury and Impaired Mitochondrial Integrity

### 2.1. Microcirculatory Reperfusion Injury

The pathogenesis of IRI involves microcirculatory injury-related no-reflow. At the molecular levels, reperfusion-triggered intracellular calcium overload, local accumulation of inflammatory cells due to blood flow restoration, excessive production of reactive oxygen species (ROS), and deficiency of high-energy phosphate compounds contribute to the development of microvascular injury [7, 18–22]. Structurally, microcirculatory disturbances are characterized by endothelial swelling, microvascular spasm, and increased capillary resistance, consequently hindering or interrupting the communication between cardiomyocyte and fresh blood flow, with an effect that is followed by increased apoptosis of myocardial microvascular endothelial cells [23–26]. Of note, both the structure and function of microvascular endothelium determine microvascular reperfusion and blood supply to cardiomyocytes [27–29]. No-reflow has been clinically observed in approximately 10% to 50% of patients with IRI.

Reperfusion causes the platelets to bind neutrophils, promotes the retention of inflammatory cells in the microcirculation [30–32], and therefore interferes with the diastolic function of the microcirculation, resulting into decreased blood flow to reperfused myocardium [33–35]. In addition, reperfusion-induced endothelial damage exposes the subendothelial collagen, allowing rapid binding of platelets to the surface of the microvascular endothelium through surface adhesion factors [36–38]. This cascade of events activates local platelets by releasing platelet factors, leading to microthrombosis and ultimately blocking the blood flow [39–41]. Although the blow flow through the epicardial large vessels is smooth, small vessels remain insufficiently perfused, causing secondary ischemia, local blood hypoperfusion, impaired energy metabolism, and consumption of high-energy phosphate compounds [9, 42].

The article "Protective Effect of Nicorandil on Cardiac Microvascular Injury: Role of Mitochondrial Integrity" was retracted in 2023. Reasons: signs of a paper mill; suspected computer-generated content; unreliable results or conclusions; concerns about the data.

Inadequate energy production limits cellular calcium recycling and contributes to intracellular calcium overload. Under physiological conditions, an appropriate increase in mitochondrial Ca^2+^ is associated with the augmented tricarboxylic acid cycle and ATP production [43–45]. Similarly, appropriate cytoplasmic Ca^2+^ levels increase cardiomyocyte contractility through calcium sparks. Besides, a moderate elevation in baseline Ca^2+^ levels improves cytoskeletal tension and endothelial motility [36, 46]. However, excessive Ca^2+^ accumulation can directly activate calcium-dependent protein kinases to trigger the endothelial apoptotic pathway. In addition, increased Ca^2+^ concentrations activate calcium-dependent xanthine oxidase (XO), inducing oxidative stress in endothelial cells [29]. The cytoplasmic calcium overload of endothelial cells, accompanied by mitochondrial calcium overload, induces cytoskeletal disintegration and impairs filamentous pseudopod formation through the IP3R- Ca^2+^-VDAC signaling pathway. These events cause impaired migration of endothelial cells and their reduced ability to revascularize after AMI [23, 47–49], ultimately causing myocardial remodeling and heart failure [41, 50–52]. Thus, abnormal calcium signals aggravate oxidative stress, trigger mitochondrial damage, destroy endothelial motility and chemotaxis, promote apoptosis, and induce endothelial reperfusion injury and microcirculation dysfunction (Table 1).

The endothelial barrier function is highly dependent on the expression of VE-cadherin that participates in endothelial filtration and resistance to substances in the blood through local gap junctions [53, 54]. IRI is characterized by reduced VE-cadherin expression, causing leakage of inflammatory cells into the subendothelial myocardium [55–57]. Although reperfusion-induced moderate inflammatory response helps to remove necrotic tissue and thus promote the reconstruction of the infarcted myocardium, excessive inflammation induces residual myocyte dysfunction, exacerbating the myocardial injury and inducing oxidative stress in the myocardium and endothelial cells [37, 58, 59].

Microcirculation damage is closely associated with augmented IRI via multiple pathophysiological processes. Oxidative stress is one of the primary features of MIRI. First, abnormal redox biology substantially consumes the levels of reduced hydrogen [60–62]. Second, excessive ROS accumulation within the cytoplasm induces oxidation of lipid components in the mitochondrial membrane, especially cardiolipin, altering the mitochondrial membrane permeability, inducing changes in mitochondrial membrane potential, and disrupting energy metabolism [63–65]. Third, overproduced ROS disrupts the endoplasmic reticulum (ER) membrane structure and interferes with the modification of proteins, consequently increasing the level of unfolded proteins and causing ER stress. Fourth, excessive oxidative stress induces the oxidation of sarco/endoplasmic reticulum Ca2 + -ATPase (SERCA), a calcium recycling protein, in the ER [29, 66], thus, reducing ER calcium recycling capacity and inducing cellular calcium overload and endothelial cell apoptosis [67] (Table 1).

The article "Protective Effect of Nicorandil on Cardiac Microvascular Injury: Role of Mitochondrial Integrity" was retracted in 2023. Reasons: signs of a paper mill; suspected computer-generated content; unreliable results or conclusions; concerns about the data.

### 2.2. Impaired Mitochondrial Integrity

Mitochondria are membrane-bound eukaryotic organelles that synthesize ATP, maintain Ca^2+^ steady-state, generate ROS, and regulate apoptosis, mitophagy, and the opening of mitochondrial permeability transition pore (mPTP) in cardiomyocytes [68, 69]. Mitochondria play a necessary role in myocardial metabolism through affecting mitochondrial dynamics, mitochondrial biogenesis, Ca^2+^ homeostasis, and redox biology [70, 71]. Myocardial ischemia is followed by mitochondrial injury, which aggravates the IRI since Ca^2+^ overload will in turn disrupt mitochondrial structure and function.

Endothelial cells contain fewer mitochondria than cardiomyocytes; they fulfill 75% of their energy demands from glycolysis rather than mitochondrial oxidative phosphorylation. Instead of serving as traditional energy centers, mitochondria in endothelial cells participate in various signal transduction as well as endothelial stress responses [63, 72–74]. Recent studies have implicated mitochondrial dynamics (mitochondrial fission, fusion, and autophagy) in maintaining mitochondrial integrity [75]. During IRI, high levels of Na^+^ activate reverse Na^+^/Ca^2+^ exchange, causing massive Ca^2+^ influx into the cytoplasm. In addition, insufficient ATP production and restoration of the mitochondrial membrane potential reduce the activity of the Ca^2+^ pump and consequently activate the activity of mitochondrial calcium uniporter (MCU), resulting into intracellular Ca^2+^ overload and exacerbating mitochondrial damage [76–78]. The initial phase of myocardial ischemia and reperfusion is characterized by an explosive increase in ROS, causing oxidative stress, lipid peroxidation, and mitochondrial damage [79–81]. Although mitophagy is able to clear the damaged cardiomyocytes and protects the adjacent normal myocardial tissues under physiological conditions [82], massive production of ROS and Ca^2+^ overload not only inhibit the activity of mitophagy but also delay the opening of mPTP, an effect that is followed by increased permeability of the mitochondrial outer membrane. The delayed opening of mPTP also induces mitochondrial swelling and membrane rupture, promotes cytochrome C (Cyt C) release into the cytoplasm [83, 84], increases Bax expression, and decreases Bcl2 expression, ultimately activating the mitochondria-dependent apoptotic cascade in reperfused heart tissues [85, 86] (Figure 1, Table 1).

The article "Protective Effect of Nicorandil on Cardiac Microvascular Injury: Role of Mitochondrial Integrity" was retracted in 2023. Reasons: signs of a paper mill; suspected computer-generated content; unreliable results or conclusions; concerns about the data.

## 3. Effects of Nicorandil on Mitochondrial Integrity

### 3.1. Dilation of Coronary Arteries

Nicorandil exerts its anti-ischemic effect primarily through dilating the coronary arteries and reducing myocardial oxygen demand. The opening of K_ATP_ channels in vascular smooth muscle cells by nicorandil hyperpolarizes the membrane, closing voltage-sensitive calcium channels and reducing the calcium inflow, ultimately reducing the vascular resistance and therefore promoting the dilation of the blood vessels [87, 88]. Furthermore, its nitrate effect generates NO free radicals, which directly activate the guanylate cyclase and increase cGMP synthesis in myocardial microcirculation. Elevated cGMP levels, in turn, target cGMP-dependent kinases and cyclic nucleotide-gated ion channel effectors [89–91]. Reduced intracellular free Ca^2+^ and desensitization of smooth muscle cell contractile proteins to Ca^2+^ result in vasodilation, decreased vascular resistance, and widening of blood vessels [92].

### 3.2. Oxidation-Resistance and Anti-Inflammation Effects

Repeated transient coronary occlusion will increase the myocardial tolerance to prolonged ischemia and reduce infarct size after myocardial infarction, which is termed by ischemic preconditioning (IPC) [93, 94]. The mitochondrial K_ATP_ (mito-K_ATP_) channel is the terminal effector of IPC. Short-term ischemia can increase the resistance of the myocardium to subsequent long-term ischemia and protect the heart by reducing oxidative stress during and after IRI [95–97]. Cardiomyocyte mito-K_ATP_ is closed at the basic state and opens at the stage of ischemia, whereas nicorandil is capable to improve myocardial resistance to ischemia challenge by opening mito-K_ATP_ channels, which enhance the cardioprotective actions of IPC. During myocardial ischemia, intracellular Ca^2+^ increases, mitochondrial matrix contracts, respiratory function is impaired, ATP production decreases, and myocardial cells become apoptotic. Nicorandil, as a K_ATP_ channel agonist, directly opens the mito-K_ATP_ channels, increases mitochondrial K^+^ inward flow, decreases the transmembrane potential difference, depolarizes the mitochondrial membrane, reduces Ca^2+^ inward flow dynamics, inhibits Ca^2+^ inward flow, and effectively prevents calcium overload in mitochondria, leading to mitochondrial relaxation, enhanced respiratory function, and increased ATP production. These regulatory effects finally protect the reperfused heart through reducing cardiomyocyte apoptosis and mitigating cardiomyocyte injury and apoptosis [16, 17, 98].

The article "Protective Effect of Nicorandil on Cardiac Microvascular Injury: Role of Mitochondrial Integrity" was retracted in 2023. Reasons: signs of a paper mill; suspected computer-generated content; unreliable results or conclusions; concerns about the data.

Inflammatory response after AMI promotes cardiac healing during IRI, whereas prolonged inflammation enhances postischemic injury and adverse cardiac remodeling [99]. Su et al. [99] constructed a coronary microembolization (CME) rat model and demonstrated that nicorandil inhibited myocardial inflammation, alleviated myocardial injury, and improved cardiac function primarily by inhibiting Toll-like receptor 4- (TLR4-) induced myeloid differentiation primary response protein 88- (MyD88-) dependent activation of nuclear factor-kappa B (NF-*κ*B) signaling pathway. These alterations reduced the release of proinflammatory cytokines, such as tumor necrosis factor- (TNF-) *α* and interleukin- (IL-) 1*β*, from ischemic cardiomyocytes. Similarly, Zhang et al. [100] showed that nicorandil maintained the macrophage M1/M2 status in M1 and M2 cell models by inhibiting the differentiation of monocytes into mature macrophages, suppressing M1 phenotype transition, and promoting the transition to the M2 phenotype to exert anti-inflammatory effects. In addition, both of their data demonstrated that NF-*κ*b and its target gene controlled the macrophage phenotype (Table 1).

Oxidative stress or redox imbalance resulting from the excessive generation of ROS during reperfusion is one of the major contributing factors to IRI pathogenesis. Some of its detrimental effects include macromolecule oxidation, membrane lipid peroxidation, membrane dysfunction, altered calcium homeostasis, neutrophil migration, DNA lesions, mitochondria-triggered apoptosis, and mPTP opening [69]. Nicorandil, as K_ATP_ channel agonists, slightly lowers the mitochondrial membrane potential and prevents ROS formation without compromising the cellular energetics during hypoxia-reoxygenation attack as well as IRI [101, 102]. Nicorandil alleviated mitochondrial Ca^2+^ overload and depolarized the mitochondrial membrane in rat ventricular cells [103]. In addition, the nicotinamide moiety of nicorandil exerted appreciable hydroxyl radical scavenging activity via a mechanism independent from its K_ATP_ channel opening effect [81, 104] (Figure 2, Table 1).

The article "Protective Effect of Nicorandil on Cardiac Microvascular Injury: Role of Mitochondrial Integrity" was retracted in 2023. Reasons: signs of a paper mill; suspected computer-generated content; unreliable results or conclusions; concerns about the data.

### 3.3. Enhanced Myocardial Ischemic Preconditioning

Pretreatment with low doses of nicorandil reduced IRI in rats by selectively opening the mito-K_ATP_ channels [105] and protected cardiomyocytes against IRI biochemical changes and ventricular arrhythmias. The use of 5-hydroxydecanoate, a mito-K_ATP_ channel selective blocker, inhibited the protective effects of nicorandil on the ventricular myocardium, confirming the function of mito-K_ATP_ on improving coronary microcirculation and protecting the myocardium [105]. Therefore, the mito-K_ATP_ channel serves as a terminal effector of myocardial IPC-short-term ischemia that increases the myocardial resistance to subsequent long-term ischemia and protects the heart by reducing oxidative stress during IRI [95, 96]. Murry et al. [96] showed that four 5-minute episodes of ischemia followed by a sustained 40-minute coronary occlusion caused less necrosis compared with a single 40-minute occlusion in the canine heart. However, this protective effect disappeared when sustained blood loss was prolonged to 3 h [88, 106]. Interestingly, nicorandil opens the mito-K_ATP_ channels to mimic or enhance myocardial IPC and therefore improve myocardial ischemic resistance (Table 1).

The glycolytic pathway serves as the primary energy production pathway under myocardial ischemia. During reperfusion, Na^+^/H^+^ exchange protein (NHE) is activated; H^+^ is transported out of the cell, and the intracellular Na^+^ increases greatly. Due to insufficient ATP produced by glycolysis to meet the normal requirements of cardiomyocytes, the activity of Na^+^-K^+^-ATP is inhibited causing Na^+^ overload (Na^+^ cannot be expelled from cells) and activating the reverse Na^+^/Ca^2+^ exchange. The abundant Ca^2+^ inward flow eventually causes Ca^2+^ overload [107–109]. Nicorandil treatment opened mito-K_ATP_ channels allowing abundant K^+^ to enter the mitochondria, hyperpolarized mitochondrial membranes, promoted K^+^-Ca^2+^ exchange, inhibited Ca^2+^ influx, and improved Ca^2+^ overload in a rabbit ischemic cardiomyocyte model [98] (Table 1).

### 3.4. Reduced Cardiomyocyte Apoptosis Caused by Ischemia–Reperfusion Injury

Mitochondria function both as the primary source of intracellular ROS generation and the regulatory center of apoptosis. Mitochondria regulate apoptosis via the main executor, Caspase-3—a member of the Caspase cysteine protease family. Cytoplasmic Cyt C interacts with apoptosis protease activating factor-1 (Apaf1) in the presence of deoxyadenosine triphosphate (dATP) and ATP and polymerizes to form apoptotic bodies. Subsequently, it activates the upstream factor Caspase-9 and the downstream factors such as Caspase-3, Caspase-6, and Caspase-7 in a cascade event, eventually causing apoptosis [110]. In addition, either Bax or Bak induces the release of Cyt C into the cytoplasm [86, 111–113]. Decreased expression of Bcl-2 increases the expression of Bax and Bak to accelerate apoptosis, whereas increased expression of Bcl-2 produces the opposite effect on reperfused hearts.

The article "Protective Effect of Nicorandil on Cardiac Microvascular Injury: Role of Mitochondrial Integrity" was retracted in 2023. Reasons: signs of a paper mill; suspected computer-generated content; unreliable results or conclusions; concerns about the data.

A surge in ROS causes oxidative stress and lipid peroxidation, whereas oxidative stress, in turn, increases ROS due to impaired mitochondrial electron transport chain (ETC) and reduced activity of antioxidant enzymes [79, 80, 114]. Ca^2+^ overload, ROS surge, and pH changes work together to open the mPTP as well as prolong its opening time by activating cyclophilin D (Cyp D), an essential component of mPTP. mPTP is a nonspecific, highly conductive, multiprotein channel located in the mitochondrial membrane gap. It remains inactive under physiological conditions, maintains ion mobility both inside and outside the mitochondria along with a stable membrane potential difference, and regulates mitochondrial membrane permeability [111]. Its irreversible opening during IRI triggers cardiomyocyte necrosis rather than apoptosis [115]. mPTP remains closed during acute myocardial ischemia and opens within the first few minutes of reperfusion, allowing small molecules, which normally cannot cross the mitochondrial membranes, to pass through, thus, increasing the osmotic pressure of the mitochondrial matrix, inducing mitochondrial fragmentation, and releasing Cyt C [83, 112, 116–118] (Figure 2).

Nicorandil-induced opening of mito-K_ATP_ channels triggers the production of low levels of ROS that are incapable of causing oxidative damage [119–121]. In contrast, elevated ROS activate several signaling pathways, stimulate mitochondrial antioxidant effect, and inhibit mitochondrial nicotinamide adenine dinucleotide phosphate oxidase—a major source of ROS production in cardiomyocytes [122]. Furthermore, nicorandil inhibits the release of Cyt C. The simultaneous increase in mitochondrial Bcl2 levels and decrease in Bax levels (elevated Bcl2/Bax ratio) inhibit the apoptotic pathway [123]. Another study showed that Bcl2 overexpression prolonged the survival time of mice, represented by reduced mitochondrial abnormalities, restored cardiac function, and decreased apoptosis [124] (Table 1). Nicorandil pretreatment reduces Ca^2+^ overload, increases ROS at a low level, enhances ATP production, inhibits ATP consumption, decreases Cyt C release, reduces mPTP opening [125, 126], shortens the ischemic PC period, and inhibits apoptotic signaling pathways, thereby ameliorating mitochondrial dysfunction and allowing better myocardial salvage during reperfusion therapy (Table 1).

The article "Protective Effect of Nicorandil on Cardiac Microvascular Injury: Role of Mitochondrial Integrity" was retracted in 2023. Reasons: signs of a paper mill; suspected computer-generated content; unreliable results or conclusions; concerns about the data.

To conclude, nicorandil improves coronary microvascular function and restores microvascular dynamics, making it one of the most promising drugs for treating CMD. However, little literature is available on it, mostly including small-scale randomized controlled trials with a few reports on its anti-CMD long-term effects. Because multiple mechanisms are implicated in CMD, combination therapy of nicorandil can prove to be highly effective [127]. With the research on the role of nicorandil in maintaining mitochondrial homeostasis, the cardiovascular protective mechanism of nicorandil has become increasingly clear and will be more and more widely used in clinical.

## Figures and Tables

**Figure 1:** Schematic representation of impaired mitochondrial integrity in microcirculatory reperfusion injury.

**Figure 2:** Schematic representation of the mechanism of nicorandil in maintaining mitochondrial integrity.

**Table 1:** Summary of studies on the protective functions of nicorandil in myocardial microcirculation.

Authors	Type of study	Models	Mechanism
Ozcan et al., 2002 [101]	Basic study	Rats	Functions as a K^+^ channel opener and directly attenuates mitochondrial oxidative stress at reoxygenation.

Ishida et al., 2004 [103]	Basic study	Rats	Attenuates matrix Ca^2+^ overload with accompanying depolarization of the mitochondrial membrane.

Ono, 2004 [17]	Clinical study		Improvement in cardiac function and clinical outcomes in patients with AMI with nicorandil may be associated with the suppression of ROS formation.

Kim, 2006 [120]	Basic study	Rats	Mitochondrial ROS promotes MPT onset and subsequent myocyte death after reperfusion.

Lu, 2006 [102]	Basic study	Rats	Nicorandil protects against postischemic left ventricular dysfunction by opening the mito-K_ATP_ channels, decreasing hydroxyl radicals, and increasing the coronary flow in the isolated rat heart.

Nishikawa, 2006 [98]	Basic study	Rats	Nicorandil regulates the Bcl-2 family proteins by opening the mito-K_ATP_ channels, induces NO-cGMP signaling, and inhibits the hypoxia-induced mitochondrial death pathway.

Tsujimoto, 2006 [108]	Basic study	Rats	Bcl-2 and Bcl-x(L) blocked MPT by directly inhibiting the VDAC activity.

Azadeh, 2009 [104]	Basic study	Rats	NO donation and free-radical scavenging properties of nicorandil may upregulate endothelial NO synthase.

Li, 2010 [123]	Basic study	Rats	DNA fragmentation is regulated by the mitochondrial fission machinery.

Maloyan, 2010 [124]	Basic study	Mice	Overexpression of Bcl-2 increases the lifespan of cardiomyocytes and ameliorates cardiac dysfunction, prevents mitochondrial swelling, and inhibits the apoptotic response in CryABR120G mice.

Ahmed, 2011 [105]	Basic study	Rats	Nicorandil (3 mg/kg) improves energy production and lowers the elevated myeloperoxidase activity.

Ahmed, 2013 [95]	Basic study	Rats	Nicorandil reduces albuminuria and ameliorates renal injury by blocking oxidative stress in chronic kidney disease.

Shahzad, 2013 [125]	Basic study	Rats	Postconditioning by hypoxia/reoxygenation prevents reperfusion injury by limiting mitochondrial Ca^2+^ load and thus opening MPTP in isolated cardiomyocytes.

Zhang, 2016 [29]	Basic study	Rats	H/R induces CMEC oxidative damage through the SR-Ca^2+^-XO-ROS injury signals.

Zollbrecht, 2016 [63]	Basic study	Rats	Nitrite-induced inhibition of NOX activity may be related to changes in NOX2 expression and XOR function.

Chan, 2017 [83]	Basic study	Rats	SIRT1 expression was repressed, acetylated p53 expression was enhanced, LOX-1/oxidative stress was upregulated in monocytes of patients with CAD, thereby increasing proapoptotic events and proinflammatory responses.

Jin, 2017 [66]	Basic study	Mice	ATF6 decreases myocardial I/R damage by linking ER stress and oxidative stress gene programs.

Zhang, 2017 [100]	Basic study	Mice	Nicorandil effectively inhibits the NF-*κ*b signaling pathway during the pathogenesis of MI by regulating the M1/M2 status and promoting angiogenesis.

Su, 2018 [99]	Basic study	Rats	Nicorandil protected cardiomyocytes from CME-induced myocardial injury primarily by inhibiting TLR4/MyD88/NF-*κ*B signaling.

Zhu, 2018 [23]	Basic study	Mice	XO-dependent oxidative damage and filopodia-related cellular migration, ultimately leading to endothelial apoptosis and migratory inhibition.

Sánchez-Duarte, 2020 [119]	Basic study	Chicken	Nicorandil affects the mitochondrial respiratory chain function by increasing the complex III activity and ROS production in skeletal muscle mitochondria.

MPT: mitochondrial permeability transition; H/R: hypoxia/reoxygenation; CMECs: cardiac microvascular endothelial cells.
